# Joint Deep-Learning-Enabled Impact of Holistic Care on Line Coagulation in Hemodialysis

**DOI:** 10.1155/2021/3413692

**Published:** 2021-12-16

**Authors:** Haisu Zhang, Wei Huang

**Affiliations:** ^1^Hemodialysis Room, Wenling Traditional Chinese Medicine Hospital, Wenling 317500, Zhejiang, China; ^2^Hemodialysis Room, Taizhou Hospital of Zhejiang Province Affiliated to Wenzhou Medical University, Linhai 317000, Zhejiang, China

## Abstract

In order to investigate the impact of holistic care on line coagulation and safety in hemodialysis and to address limitations of the conventional ultrasound flow vector imaging (VFM) technique, which requires proprietary software to acquire raw Doppler and scatter tracking data, a combined deep-learning-enabled holistic care approach to line coagulation in hemodialysis is proposed. First, velocity along the direction of the sound beam, which is provided by the color Doppler echocardiogram, is obtained as the radial velocity component using a velocity scale. Moreover, the left ventricular wall contour is automatically identified using a U-Net network and the left ventricular wall velocity is calculated as the boundary condition of continuity equation by a retrained PWC-Net model. Likewise, the velocity component of each blood mass in the vertical direction of the sound beam is obtained by solving the continuity equation (i.e. tangential velocity component). Finally, the velocity vector map of cardiac flow field was synthesized and visualized in the flow diagram. For this purpose, sixty patients admitted to receive hemodialysis from February 2019 to June 2020 were randomly divided into two groups of 30 patients where the control group implemented conventional care and the study group implemented all-round care on the basis of conventional care. The nursing effects of both groups were compared. Incidence of pipeline coagulation and complications in the study group were lower than those in the control group and the difference was statistically significant (*P* < 0.05). The nursing detail score, nursing attitude score, nursing professionalism score, and total satisfaction score in the study group were higher than those in the control group and the difference was statistically significant (*P* < 0.05). Applying all-round nursing in hemodialysis can effectively reduce the incidence of line coagulation complications and improve the safety of hemodialysis, as well as improve patients' satisfaction with nursing care.

## 1. Introduction

Hemodialysis is among the main protocol for clinical treatment of uremia, which is mainly used to remove the patient's organism. The main purpose of hemodialysis is to correct the water-electrolyte and acid-base balance of the patient by removing the retained substances to maintain the normal metabolism of the body, improve the quality of survival, and prolong the survival period of the patient [1]. The treatment process of hemodialysis is complex, and if care is not appropriate, then it is very easy to produce safety risks. Additionally, due to the influence of many factors, line coagulation is more common in hemodialysis, and if line coagulation or other safety risks occur, it will not only reduce the quality of hemodialysis treatment, but also threaten the life safety of patients [2]. Therefore, in hemodialysis care, it is important to prevent line coagulation and improve dialysis safety. However, conventional care in the past could not take into account all aspects of the patient, which increased the safety risks of hemodialysis to a certain extent. As a nursing model that emphasizes all aspects of care, comprehensive care has been widely used in hemodialysis patients in recent years, and its nursing effect has been recognized by many medical practitioners [3].

Cardiovascular disease is a serious threat to human health in daily life, and its incidence and mortality rate have always been the highest. According to the World Health Organization (WHO), cardiovascular disease kills approximately 17 million people worldwide each year, accounting for 31% of all deaths worldwide. The reason why cardiovascular disease has such a high mortality rate is that there are usually no obvious clinical manifestations in the early stages of cardiovascular disease. Therefore, the key to prevention and treatment of heart disease is early detection and early treatment. In fact, the morphological structure and blood flow pattern of the heart are already different from those of normal people in the early stage of the disease, and the abnormalities of cardiac function can be reflected in a timely and effective manner by observing the changes in the hydrodynamic state of the heart [1]. Therefore, effective visual observation and quantitative evaluation of cardiac hydrodynamic motion state can help early screening of cardiac function abnormalities and provide a new technical means for early detection of cardiovascular diseases.

Ultrasound has the advantages of being noninvasive, radiation-free, real-time, inexpensive, and simple to operate. Therefore, ultrasound imaging techniques have been widely used in clinical practice for visualizing and measuring blood flow, such as continuous Doppler, pulsed Doppler, and color Doppler. However, these methods can only reflect the partial information of the flow field to a certain extent but cannot fully reflect the fluid motion state. The emergence of VFM has enabled the visualization of the whole flow field of the heart, especially in the visualization of left ventricular motion and quantitative evaluation studies, which was first proposed by Ref. [2] as a novel technique for the detection of cardiac function. A three-dimensional numerical model for the validation was presented, but its flow field velocity estimation method had theoretical shortcomings [3]. An improved method combining ventricular wall motion information with Doppler velocities to obtain a valid LV flow field velocity vector is presented [4]. Likewise, a model-based improvement of weight division was presented in [4] to obtain an effective LV flow field velocity vector. Moreover, a calculation mechanism is provided in [5] to improve the weight division, which is based on Garcia. Authors have computed the Doppler flow function by extending the flow function and finally achieved a visual description of the two-dimensional planar fluid motion [6]. Accuracy of VFM, both qualitatively and quantitatively, in a three-dimensional left ventricular blood flow field, are validated by comparing VFM with blood flow measurements from particle image velocimetry [7]. A new method called a posteriori VFM accuracy estimation improved the clinical validity of VFM [8]. A YLO deep learning model was integrated or combined with an improved block matching algorithm to localize and track the left ventricular wall and improve the weight function to improve the accuracy of VFM [2]. However, because the existing VFM technique relies on specific ultrasound equipment to obtain raw RF data and commercial scatter tracking software before flow field visualization analysis, and requires manual outlining of the left ventricular wall during the calculation, it is not general enough and has limitations and nonportability.

In this paper, a color Doppler echocardiographic image of blood flow information to extract cardiac left ventricular flow field information from the perspective of digital image processing in conjunction with a deep learning network model is presented. Compared with existing VFM methods, the main improvements of this paper include

- Not relying on a specific ultrasound device to derive original RF signal to extract Doppler velocity information.
- Directly using any ultrasound device capable of deriving color Doppler echocardiograms.
- To obtain velocity information based on image data by breaking limitations of ultrasound devices.
- Using the U-Net model to automatically identify left ventricular wall contours, and using the PWC-Net model instead of the U-Net model to automatically identify the LV wall contour. Also, the PWC-Net model is used to estimate the displacement of the identified LV wall, which reduces the time consumption and improves the computational efficiency.
- This paper establishes a fast and generalized VFM method based entirely on image information that does not require any vendor technical support or proprietary software to accelerate the application of VFM in the clinical workflow. Based on this, 60 patients undergoing hemodialysis in the hospital from February 2019 to June 2020 were selected for this study with the aim of investigating the impact of holistic care on line coagulation and safety in hemodialysis.

The remaining paper is organized as follows:

In Section 2, working mechanisms or the proposed methodology is described along with sufficient information. In Section 3, detailed explanation and evaluation of various results is presented, which is followed by a comprehensive discussion. Lastly, concluding remarks are given.

## 2. Proposed Methodology (VFM Method)

The proposed VFM method, which is entirely based on two-dimensional color Doppler echocardiographic image information, uses a velocity scale to extract the radial velocity along the direction of the acoustic beam instead of acquiring the Doppler velocity from the raw RF data of a specific device as the radial velocity. Two deep learning networks are used to identify the left ventricular wall position and acquire the ventricular wall velocity, according to the correlation between the motion pattern of the anterior and posterior walls of the left ventricle and the fluid motion of the heart. The tangential velocity components of each blood mass in the cardiac flow field are calculated based on the correlation between the motion pattern of the anterior and posterior walls of the left ventricle and the fluid motion of the heart. In this paper, we mainly use velocity vector diagrams and planar flow diagrams to visualize the left ventricular fluid motion, reflecting the flow trend, velocity distribution characteristics, and overall blood flow structure.

### 2.1. Extraction of Radial Velocity

Color Doppler flow information contains information about the direction of blood flow movement, i.e., blood flow toward the direction of the probe is shown in red, and blood flow away from the direction of the probe is shown in blue. At the same time, color Doppler flow information contains information about the change of blood flow velocity, i.e., the higher the color brightness, the higher the velocity along the ultrasound beam direction, and the lower the color brightness, lower the velocity along the ultrasound beam direction.

The extraction of Doppler velocities from the colored blood flow information in the method proposed in this paper is a crucial step in the further study of left ventricular fluid motion. In this paper, the velocity extracted from the color blood flow information is used as the radial velocity, which becomes the first velocity component in the final formed flow field. To obtain this velocity information, the velocity scale generated on the color Doppler echocardiogram is used as a metric for measuring the velocity values. The best match between the blood masses in the color Doppler image and the velocity scale is searched by color-coding the color flow information corresponding to each blood mass, and the least squares method is used to calculate the similarity between the two:

(1) $$\begin{array}{c} c=\sqrt{{\left(R_{b}-R_{s}\right)}^{2}+{\left(G_{b}-G_{s}\right)}^{2}+{\left(B_{b}-B_{s}\right)}^{2}}, \end{array}$$

where *c* denotes the similarity between the blood plasmas and the points in the velocity scale; *R*_*b*_, *G*_*b*_, *B*_*b*_ represent the RGB color tristimulus of the currently calculated blood plasmas, and *R*_*s*_, *G*_*s*_, *B*_*s*_ represent the RGB color tristimulus of the points on the velocity scale, respectively. This step is mainly to find the optimal matching point position of the current blood mass in the velocity scale and to obtain the distance parameter of the point on the velocity scale. Then, using the segmented linear function of radial velocity versus distance [9] (as in Figure 1):

(2) $$\begin{array}{c} V_{r}\left\{\begin{array}{cc} \frac{\left(d-d_{1}\right)}{\left(-d_{1}/V_{\max}\right)}, & \text{if }0\leq d\leq d_{1},\\ \left(d-d_{2}\right)\times \frac{V_{\max}}{\left(d_{\max}-d_{2}\right)}, & \text{if }d_{2}\leq d\leq d_{\max}. \end{array}\right. \end{array}$$

In equation (2), *d* represents the pixel distance between the best match point and the bottom of the blue area of the speed scale, *d*_1_ represents the pixel height of the blue area of the speed scale, *d*_2_ represents the sum of *d*_1_ and the pixel height of the black area of the scale, *d*_max_ represents the pixel height of the entire speed scale, and *V*_max_ represents the maximum speed in the current speed scale measurement range.

The radial velocity values obtained by the velocity scale are not smooth and cannot satisfy the subsequent solution of the continuity equation. To ensure a more stable integration environment, the radial velocity data are smoothed after the original radial velocity is found using the velocity scale. The smoothing method includes median filtering and Gaussian filtering of the radial velocity data. The median filtering method is shown in Figure 2(a). For the radial velocity of the currently requested blood mass, the radial velocity value of the previous blood mass as well as the radial velocity value of the next blood mass is located along the ultrasound beam direction, and the median value of the three blood masses is obtained as the radial velocity value of the current blood mass, taking the value inside the solid coil in Figure 2(a) as an example. The Gaussian filter is processed as shown in Figure 2(b), and the window size of 5 × 5 Gaussian template (as the red box in Figure 2(b)) is generated by the two-dimensional Gaussian function (see equation (3)), and the radial velocity of the same window size range (as the black box of the same size in Figure 2(b)) centered on the current blood mass (as the red point in Figure 2(b)) is convolved, and the calculation result is taken as the current blood mass. This operation is repeated until the calculation of all blood masses is completed. The median filtering method can eliminate abnormal velocity values, and the Gaussian filtering method eliminates small-scale velocity fluctuations.

(3) $$\begin{array}{c} G\left(x,y\right)=\frac{1}{2\pi \sigma }e^{-x^{2}+y^{2}/2\sigma^{2}}, \end{array}$$

where *G* denotes the Gaussian template matrix, *s* denotes the standard deviation, which is set to 8 in this paper, *e* denotes the natural base, *y* denotes the two-dimensional position coordinates of the template, and since the template size is set to 5 × 5 in this paper, *x*, *y* = [−2, −1,0,1, 2].

### 2.2. Calculation of Tangential Velocity of Ventricular Fluid

#### 2.2.1. Calculation of Weighting Function

Using the weight function *w*, the two solutions of the linearly combined continuity equation, the final tangential velocity can be obtained as follows:

(4) $$\begin{array}{c} V_{\theta }=\left(1-w\right)V_{\theta }^{-}+wV_{\theta }^{+}. \end{array}$$

The contribution of the first solution (equation (3)) and the second solution (equation (4)) to the tangential velocity of the final blood mass is considered to make the two solutions account for a reasonable proportion of the final tangential velocity as uniformly as possible and to reduce the error of the results. The angular distance ratio is used to define the weight function:

(5) $$\begin{array}{c} w=\frac{\theta -\theta_{-}}{\theta_{+}-\theta_{-}}. \end{array}$$

That is, the ratio of the angular difference between the blood mass and the anterior wall of the left ventricle and the angular difference between the posterior wall of the left ventricle and the anterior wall of the left ventricle in the polar coordinate system is used as the weight value.

#### 2.2.2. Calculation of Tangential Velocity

Studies [5, 8, 10] have shown that the state of ventricular wall myocardial motion is closely related to cardiac disease and that abnormal motion of the ventricular wall will directly lead to changes in the hemodynamic characteristics of the cardiac chambers. Therefore, it is valuable to incorporate the motion of the ventricular wall in the study of hemodynamic characteristics. In this paper, we use temporal resolution reconstructed color Doppler images to be analyzed after pulmonary echocardiographic image and its adjacent posterior color Doppler echocardiographic image, and the left ventricular wall contour is automatically identified using the U-Net deep learning framework. After taking the identified LV wall contours, a retrained PWC-Net model is used to estimate the pixel displacement. The final physical tangential velocity of the left ventricular wall is obtained using the temporal resolution set by the ultrasound device and the position information of the ventricular wall, which is used as a boundary condition for the continuity equation.

### 2.3. Automatic Ventricular Wall Contour Recognition Method

Most of the existing studies on LV flow vector imaging techniques use a semi-automatic method of manual outlining by clinicians or manual outlining combined with automatic identification to identify LV wall contours [3, 4, 7, 8]; they often rely on the clinical experience of physicians to make judgments, which is highly subjective, and such a manual method, although accurate, affects the efficiency of the calculation, and different physicians' outlines of left ventricular wall position can also differ, which can have an impact on the calculated flow field results.

In this paper, we use the deep learning method to implement automatic segmentation recognition function of left ventricle contour. For medical images, the U-Net network model shows better segmentation performance. The U-Net model [11] is a codec structure, and the codec structure of the network is very suitable for segmentation. The U-Net network follows a specific approach in which each down-sampling step and up-sampling step goes through two 3 × 3 convolutional layers, while the number of features for each down-sampling process is doubled compared to the number of features for the up sampling. The number of features in each down-sampling process is doubled and the number of features in the up-sampling process is halved. Specifically, the left half of the model is the down-sampling process and the right half is the up-sampling process. The-down sampling process mainly passes through successive 3 × 3 convolutional layers with a Re LU activation layer and a 2 × 2 maximum pooling layer, continuously extracting image features up to the highest dimension. The up-sampling process maps the higher features to the lower dimension by successive 2 × 2 up convolution, and connects the corresponding cropped image features from the down-sampling process to obtain the classification of each pixel in the image and output the segmented image, which is shown in Figure 3.

In this paper, we use the largest and publicly available fully annotated CAMUS dataset for 2D echocardiographic evaluation [2]. This dataset is a large dataset with full-label annotation, containing 10 folders, each containing 50 patients with ultrasound acquisition sequences of at least one cardiac cycle in 2D B-mode, as well as end-diastolic and end-systolic two-chamber and four-chamber images and their corresponding endocardial (i.e., LV wall), LV epicardial, LV, and background four-chamber images annotated by three cardiac disease experts under a protocol, atrium, and background four labels.

The region of interest, specifically in this paper, is the region of the left ventricular wall, and the location of the left ventricular wall needs to be identified as the boundary condition of the continuity equation. In order to improve the speed of training, this paper preprocesses the labels of the original dataset, only the left ventricular endocardium and background labels are preserved, and the U-Net model is used to train the left ventricle for binary classification.

In the actual model training process, Keras was used as the deep learning framework, and data from a total of 400 patients in 8 folders (1,600 images in total) were used as the training set, and data from a total of 50 patients in 1 folder (200 images in total) were used as the test set. According to the method proposed in this paper, the training parameters were finally determined after extensive experimental training for the recognition needs of the left ventricular wall contour: to obtain higher dimensional feature maps, convolutional and maximum pooling layers were used in the down-sampling path until the feature dimension was 16 × 16; the batch normalization method was used; the batch size was set to 2; the learning rate was set to 1*e* − 04; the stochastic gradient descent method was used as the optimization strategy; and the loss function is cross-entropy and regularization. The final segmentation model of the left ventricular wall was obtained.

#### 2.3.1. PWC-Net Optical Flow Network Calculation of Chamber Wall Motion

The idea of the PWC-Net model is very close to the multi-scale optical flow method. The structure of the model is shown in Figure 4. In the *i*th scale, the PWC-Net model first extracts the image features from the two input images *I*_1_ and *I*_2_, which can be denoted as *f*_*i*1_^*i*^ and *f*_*i*2_^*i*^, and uses the up-sampled displacement estimates from the previous scale (i.e., the (*i* − 1) scale) and convolves *f*_*i*2_^*i*^ as motion compensation features, denoted as ${\tilde{f}}_{I2}^{i}$. Then, after matching ${\tilde{f}}_{I2}^{i}$ and *f*_*i*1_^*i*^ into pairs, the displacements are estimated using a multilayer CNN. After the CNN, an optional contextual network layer (an additional convolutional layer) is included that can be used to further optimize the displacement estimates. The entire training process is repeated for scale *i* until the process is performed for all scales, resulting in the output displacement data.

Since cardiac motion is a free-form nonrigid motion process, the training of the original PWC-Net optical flow network model is done by natural image data, so this paper uses the finite element software ANSYS and ultrasound simulator Field II to generate the ultrasound nonrigid motion dataset. The resulting displacements were retained and added to the pre-compression tissue model for obtaining post-compression images, and then the pre- and post-compression tissue models were imaged by ultrasound simulation on the Field II platform to obtain B-mode ultrasound image pairs before and after compression. The simulated ultrasound datasets include four small spherical mimicry data pairs before and after compression and complex breast structure data pairs before and after compression, and the information of the datasets is shown in Table 1.

A new PWC-Net model was obtained by migration learning of the original PWC-Net model using the shifts retained by the simulated data as labels and simulated B-mode ultrasound image pairs as the training set [12], and the model was initialized with the original PWC-Net model parameters during the training process, and four small ball mimic data were involved in the first stage of migration training of the model. After convergence of the model, the PWC-Net network is initialized with the model obtained in the first stage, and the complex breast mimic data are used for the second stage of migration training of the model. The important training parameters of the model are shown in Table 2, where *S*_long_, *S*_fine_ are consistent with the description in the literature [9], and the first stage is the coarse training stage, and the L2 loss is chosen as the loss function, which has a fast convergence rate and a stable solution to control the complexity of the model. The second stage is the fine training stage, where L1 loss is chosen as the loss function, which has better robustness to deal with the outliers in the simulated data [13].

In this paper, the cropped left ventricular region of the current image frame and the corresponding region of the adjacent next image frame are used as input images, and the displacement of the whole left ventricular region, including the horizontal pixel displacement and the vertical pixel displacement values, is finally obtained using the retrained PWC-Net model. Then, using the U-Net trained in the paper model obtained in this paper, only the displacement data of the left ventricular e-wall are retained, and the physical tangential velocity of the left ventricular wall can be obtained by using the time interval between image frames set at the time of ultrasound device acquisition and the angular position of the requested ventricular wall point on the polar coordinate system.

### 2.4. Steps of the Proposed Method

Steps of the visual description method in this paper are as follows:

  Input: Color Doppler echocardiogram
  Output: Velocity vector and streamline visualization results
  Step 1: Rational selection of images of typical phases in the cardiac cycle; two sets of experimental images were selected in this paper, and two sets of experimental images were in the systolic phase. Crop out the left ventricular range as the region of interest.
  Step 2: Supplement the colored blood flow information at the gaps in the region of interest using a one-dimensional linear interpolation method.
  Step 3: Extract the radial velocity components of all the blood masses in the region of interest using the velocity scale and smoothing, which includes median filtering and Gaussian filtering.
  Step 4: Automatically identify the left ventricular wall location using the trained U-Net model and reconstruct the image sequence to improve temporal resolution.
  Step 5: Solve the tangential velocity of the left ventricular wall using the retrained PWC-Net deep learning model.
  Step 6: The tangential velocity components of all blood masses in the left ventricular region are obtained by the calculation of equation.
  Step 7: The radial velocity component and tangential velocity component are obtained to synthesize the blood flow velocity field, the velocity vector diagram is drawn to observe the characteristics and magnitude of the blood velocity distribution, and the flow line diagram is drawn on the basis of the velocity vector diagram to observe the blood structure characteristics of the fluid in the left ventricular chamber.

The specific algorithm flow is shown in Figure 5.

## 3. Experimental Results and Analysis

In this section, we have briefly analyzed various results obtained through sophisticated experiments on different patients in the hospitals.

### 3.1. Data Acquisition

Sixty patients admitted to receive hemodialysis, specifically from February 2019 to June 2020, were randomly divided into two groups of 30 cases each. In the control group, there were 18 males and 12 females; ages ranged from 30 to 71 years, with an average of 50.39 ± 5.37 years; education level: 3 cases in elementary school, 5 cases in junior high school, 10 cases in high school or junior college, 7 cases in college, and 5 cases in undergraduate level and above. In the study group, there were 16 males and 14 females; ages ranged from 28 to 70 years, with a mean of 50.31 ± 5.30 years; education level: 4 cases in elementary school, 6 cases in junior high school, 11 cases in high school or junior college, 5 cases in college, and 4 cases in undergraduate level and above. The study was approved by the ethics committee. The general data of the two groups of patients were compared, and the differences were not statistically significant (*P* > 0.05) and were comparable. Inclusion criteria: diagnosed uremia by laboratory examination and hemodialysis time >6 months; serum calcium ion >1.0 mmol/L; both patients and family members signed the informed consent.

Exclusion criteria: anticoagulant drugs used within the last 1 month; combined coagulation dysfunction; psychiatric (iii) mental illness.

Methods: (1) Conventional care was implemented in the control group, that is, before treatment, patients were given instructions on the precautions to be taken during treatment and the operation of the relevant equipment. During the dialysis process, nursing staff were required to closely observe the patients' vital signs, and if equipment alarms were found, they were required to immediately troubleshoot to ensure that dialysis was carried out normally. (2) The study group implemented comprehensive care on the basis of conventional care. Environmental intervention: The hemodialysis room is the main place for hemodialysis, so nursing staff should keep the hemodialysis room well-lit and airy, strengthen indoor disinfection, and change bedsheets regularly. At the same time, an escort lounge is set up for the patient's family members, and a small manual of knowledge about hemodialysis is placed in the lounge. All-round care before dialysis: (a) Psychological intervention: The influence of factors such as long duration of disease and long-term treatment leads to negative situations such as negativity, anxiety, and depression in hemodialysis patients in general. In order to ensure the smooth progress of dialysis, the nursing staff need to encourage patients and organize regular patient exchange sessions to help patients establish treatment confidence and eliminate their negative emotions.

At the same time, knowledge related to hemodialysis can be explained through lectures, and patients can be taught methods of self-regulation so that they can maintain a good state of mind. (b) All-round body assessment: Before starting hemodialysis, the nursing staff accurately measure the patient's heart rate, blood pressure, etc., while correcting water-electrolyte and acid-base disorders in a timely manner, and then start hemodialysis after the patient's body condition is stable. ③ All-round care during dialysis: (a) Puncture intervention: When performing puncture operation, the nursing staff should strictly follow the principle of aseptic operation, and the puncture action needs to be gentle to reduce the patient's pain. At the same time, on close observation after puncture, if blood leakage is found, timely treatment is required. (b) Monitoring of signs and observation of equipment: Closely observe the changes in the patient's heart rate and blood pressure, and check whether the pipeline slips and folds during the dialysis process. The patient's blood flow, blood line pressure, dialysate concentration, and temperature were observed regularly, and the patient was asked whether there was discomfort. (c) Catheter intervention: During the dialysis process, the nursing staff should ensure that the catheter drainage is smooth, and after the catheter is used, it has to be sealed with positive pressure, strictly disinfected, the heparin cap should be replaced in time, and finally the catheter mouth should be closed with sterile gauze. (d) Internal fistula intervention: Strictly control the intake of water. The weight gain between dialysis sessions should not exceed 5% of the dry weight. Prevent hypotension, perform dialysis on time, do not reduce the number of dialysis sessions or the duration of dialysis without permission, and preferably choose to eat during the pre-dialysis period. Prevent endovascular infection by keeping the skin of the arm clean and avoid contact with water at the puncture site on the last day of dialysis to prevent infection. The arm on the side of the internal fistula should not be subjected to prolonged pressure, the sleeves should be loose, holding heavy objects should be avoided, and it is forbidden to measure blood pressure, infusion, intravenous injection, and draw blood on the arm on the side of the internal fistula. Patients should learn to self-judge whether the arteriovenous endovascular fistula is open or not, that is, touch the anastomosis on the operated side with the nonoperated side of the hand; if you feel tremors, it means it is open, if the tremors and murmurs disappear and there is tenderness or pain at the fistula, you should go to the hospital in time. Avoid trauma to the arm on the side of the fistula; it is best to wear wrist guards, but wrist elasticity should be moderate, very tight compression of the intravenous fistula is to be avoided to prevent blockage of the fistula, and if there is an aneurysm, it should be protected by elastic bandages to ensure the smooth flow of blood to the fistula. ④ Post-dialysis all-round care: After the end of dialysis, perform a thorough hemostasis of the puncture site and observe whether the patient has hypotension or arrhythmia. Blood samples are to be collected for biochemical testing, and the selection of the arteriovenous endovascular limb is prohibited for blood sample collection. Patients are instructed to wear loose clothing, and their diet needs to be low-fat, low-salt, and easy to digest, with strict restriction of water intake. For patients with anemia, iron and folic acid supplements should be given. Pipeline coagulation prevention intervention: (a) The patient's coagulation status should be comprehensively assessed before dialysis treatment, and reasonable selection and application of anticoagulants is the key to prevention. For patients with hypercoagulation, the patient's coagulation function needs to be tested before dialysis to accurately calculate the amount of heparin, and the patient's venous pressure, dialyzer, and blood color in the pipeline should be closely observed. (b) Avoid the input of blood, blood products, and fatty milk during dialysis, especially the input of coagulation factors. (c) Monitor vascular access blood flow regularly to avoid recirculation expansion during dialysis. Insufficient blood flow is mostly caused by poor catheter drainage; therefore, if the catheter is poorly drained, the patient should be assisted to adjust the position; if the insufficient blood flow is not improved, thrombosis is considered, and urokinase blocking is needed regularly to prevent catheter coagulation. (d) In heparin volume intervention, the nursing staff need to accurately calculate the heparin volume intervention; they should accurately calculate the heparin injection volume, and strictly carry out “three checks and seven pairs” after getting on the machine to prevent the occurrence of pipeline coagulation (shown in Tables 3 and 4).

Observation index: Compare the incidence of line coagulation, complication rate, and nursing satisfaction scores between the two groups of patients. Complications included bleeding, catheter infection, and left heart failure. The nursing satisfaction score was investigated using our homemade nursing satisfaction scale, including three dimensions of nursing staff's nursing details, nursing attitude, and nursing professionalism, with the first two having scores of 30 each and the third having a score of 40, totaling to a score of 100, with higher scores indicating higher nursing satisfaction.

Statistical treatment: Data were processed using SPSS 22.0 software; count data were expressed as [*n* (%)] using the *χ*^2^ test; measurement data were expressed as ($\bar{x}\pm s$) using the *t*-test; *P* < 0.05 was considered a statistically significant difference.

Comparison of the incidence of line coagulation and complication rate between the two groups: The incidence of line coagulation in the study group, and the difference was statistically significant (*P* < 0.05). Comparison of nursing satisfaction scores between the two groups: Nursing detail score, nursing attitude score, nursing professionalism score, and total satisfaction score in the study group were significantly higher than those in the control group, and the difference was statistically significant (*P* < 0.05). See Table 2.

### 3.2. Data Processing

#### 3.2.1. Reconstruction of Color Doppler Echocardiographic Image Sequences

Usually, the temporal resolution of color Doppler echocardiography is not high, and the image frame rate is about 30 fps; in this case, the time interval between adjacent frames of the acquired images is long, which directly leads to the weak correlation between adjacent image frames, and the final ultrasound image sequence obviously cannot meet the requirements of subsequent ventricular. The final ultrasound image sequence obviously cannot meet the requirements of subsequent ventricular motion tracking calculation and analysis. Therefore, in order to obtain ventricular wall motion information, the temporal resolution of color Doppler echocardiography must be improved.

In this paper, based on the idea of temporal super-resolution reconstruction, multiple cardiac cycle images are reordered according to the ECG temporal phase position information in the color Doppler echocardiogram, and the images in the subsequent cardiac cycles whose temporal phases are between the corresponding adjacent frames in the first cardiac cycle are searched, and the searched images are inserted into the corresponding adjacent frames until all the adjacent frames in the first cardiac cycle are inserted by the subsequent frames. The images of the first cardiac cycle are inserted into the corresponding adjacent frames until all the adjacent frames of the first cardiac cycle are inserted by the images of the subsequent cardiac cycles.

In this paper, we use the color Doppler echocardiographic image sequence information of three cardiac cycles to obtain a new color Doppler ECG sequence with 3 times the temporal resolution of the original image by reconstruction, which ensures the computational conditions of ventricular wall motion displacement estimation.

#### 3.2.2. Color Blood Flow Information Compensation

The conventional color Doppler echocardiography imaging technique in clinical diagnosis is based on the principle of pulsed Doppler, which uses the signal of frequency shift in Doppler to obtain information on the average velocity of blood flow in the sampling area and velocity variation, and performs color Doppler encoding processing, and the color blood flow information formed is superimposed onto a two-dimensional B-mode gray-scale image to constitute a complete ultrasound color Doppler image. During the acquisition of cardiac Doppler images, low blood flow velocities in certain regions of the left ventricle of the heart can result in dim or even no color flow information after encoding. The use of velocity scales to extract radial velocities is insensitive to these low velocity regions, resulting in the loss of radial velocity details of some of the blood flow, which may make the final flow field results discontinuous.

Therefore, it is necessary to compensate some important color flow information in the original color Doppler cardiac images based on the original color flow information, so as to obtain a richer and more accurate flow field information. In this paper, we use the one-dimensional linear interpolation method to compensate the color flow information in the original image data, and the main compensation area is the gap between two different colors of color flow information, and the formula of the one-dimensional linear interpolation method is as follows:

(6) $$\begin{array}{c} y=\left(1-k\right)\times y_{0}+k\times y_{1}, \end{array}$$

where *y* represents the color value of a blood mass with no or dimly colored blood flow information, *y*_0_, *y*_1_ represents the color value of the left and right nearest blood masses containing colored blood flow information, respectively. *k* represents the ratio of the distance from the currently requested blood mass to the left neighboring blood masses containing blood flow information to the currently requested blood mass to the right neighboring blood masses containing blood flow information. The ratio of distance from the currently requested blood mass to the neighboring blood mass on the left and right contains blood flow color.

### 3.3. Original Image Color Information Supplement Results

Figures 6(a) and 6(b) belong to the intracardiac cycle images of a subject in the period typical for clinical analysis of the heart-diastole. The upper right corner of each set of test images shows the supplementary result maps corresponding to the colored blood flow information. As can be observed from the results of the two test image sets, according to the one-dimensional linear interpolation method, the colored blood flow information compensated by the colorless region is brighter the closer the points are to the colored region, and the velocity is larger relative to the points away from the colored region, which can reasonably and effectively compensate part of the colored blood flow information at the gap between the red region and the blue region. This compensation result provides a more subsequent analysis of the blood flow field in the left ventricular cavity complete information.

### 3.4. Ventricular Wall Motion Tracking Results

Figure 7 shows the comparison between the original PWC-Net and the retrained PWC-Net model for tracking the ventricular wall motion in the left ventricular region of the color Doppler echocardiogram. The comparison of transverse displacement and longitudinal displacement is formed by Figures 7(a) and 7(b) where the direct use of the original PWC-Net model for the test data shows severely stratified curves with noise, as shown in the black boxes in Figures 7(a) and 7(b), while the retrained PWC-Net shows more stable and smooth prediction results with continuity, showing that the retrained PWC-Net model can accurately estimate the motion of the left ventricular wall.

The effectiveness of the retrained PWC-Net model for nonrigid motion detection of the heart was verified by the displacement estimation results, and the retrained PWC-Net model can compute frame rates up to 45 FPS compared to the traditional nonrigid aligned motion estimation that relies on iterative solving, meeting the demand for real-time imaging.

### 3.5. Blood Flow Velocity Vector Diagram

From the two sets of velocity vector diagram results, the trend of blood movement in the left ventricular cavity and the distribution of the magnitude of blood flow velocity can be effectively observed. Figures 8(a) and 8(b) correspond to the velocity vector diagram results in Figure 8(a).

In the velocity vector diagram of Figure 8(a), the velocity of blood flow in the left ventricular cavity is higher on the inflow tract side, the blood flow touches the ventricular wall of the apical segment toward the apical position, and the direction of blood motion is shifted toward the outflow tract position.

It can be observed in the velocity vector plot of Figure 8(b) that the phase of this set of color Doppler cardiograms corresponding to the cardiac cycle is slightly later than the diastolic phase of Figure 8(a). In the velocity vector results of Figure 8(b) it can be observed that compared to the velocity vector of Figure 8(a), a large amount of blood flow steering is completed after the transapical position and the overall blood flow velocity distribution is more distant from the apical position and closer toward the basal segment of the left ventricle. The overall velocity is uniform and slightly lower on the inflow tract side compared to Figure 8(a).

Comparing the blood flow vector imaging method proposed in this paper with the post-processing analysis method of Aloka VFM workstation, it shows that the results of the two methods have a high degree of consistency, and the velocity flow field in the blood flow region shows reasonable blood flow motion trends and blood flow velocity magnitude distribution in the two sets of test images, which can effectively observe the left ventricular velocity distribution and the movement direction of blood flow velocity.

### 3.6. Plan Flow Diagram

Based on the velocity vector plotting, the results of the planar flow diagram are helpful to visualize the structural pattern of the movement of blood flow in the left ventricle more. Figures 9(a) and 9(b) correspond to the results of planar flow diagrams of Figures 8(a) and 8(b), respectively. By visualizing the flow line diagrams, the method in this paper enables to clearly observe the vortex structure in the left ventricle. The vortex structure is one of the important indicators of hemodynamics and provides more direct evidence for the auxiliary diagnosis of cardiac diseases.

In Figure 9(a), the vortex state of the blood imaged during this cardiac cycle phase can be observed. A smaller vortex appears at the location of the ventricular wall close to the inflow tract side and a larger vortex structure is formed on the side close to the outflow tract (where the red arrow points). This kinetic feature corresponds to the characteristics of human heart motion. At this stage, the blood flow collides with the ventricular wall of the apical segment of the left ventricle turning so that a larger vortex state is formed.

In Figure 9(a), a large vortex is visible to the naked eye filling the entire left ventricular cavity (indicated by the yellow arrow). At the same time, a smaller vortex appears at the location of the ventricular wall near the inflow tract side. The vortex does not disappear and remains rotating from Figures 9(a)to 9(b). The left ventricular blood is transmitted and steered by the kinetic energy of the vortex, providing sufficient kinetic support for the onset of systole.

Comparing Figure 9(a) with Figure 9(b) by visual observation analysis, the blood vortex motion states are similar, i.e., both the method proposed in this paper and the method provided by the Aloka VFM workstation are able to detect larger vortices near the outflow tract side and smaller vortices near the inflow tract side.

## 4. Discussion

Hemodialysis is a kind of blood purification technology, which mainly uses the principle of semi-permeable membrane to remove all kinds of harmful substances and excess metabolic wastes from the body in order to purify the blood and correct water-electrolyte and acid-base disorders. Presently, hemodialysis is the main treatment option for patients with uremia, and it plays an important role in prolonging the survival of patients. However, because the treatment cycle of hemodialysis is phased and long term, the physiological and psychological burden of patients increases as the number of hemodialysis sessions increases, and the treatment process of hemodialysis is very complicated, which highlights the safety risks during the treatment process. Specialized courses, distribution of relevant teaching materials, and creating awareness among students about CPR motivate them to learn CPR [2, 8].

Establish a training system: Schools should conduct targeted training, enrich the training model, standardize the training content, and establish a good training system. Content for standardization, the establishment of a good training system: Schools should develop training content according to students' mastery of CPR, focus on the implementation of low mastery knowledge, determine the training pathways according to students' capabilities, add CPR-related knowledge to the curriculum system, focus on training students at college, conduct hands-on assessment during training, which can be completed after passing; on this basis, the school should build online and offline training framework, and develop an assessment method to improve and establish a good training system [9].

Establishing cooperation mode: School hospital + college, nurse + classroom cooperation mode can be constructed for training; school hospital is an important resource for cardiac resuscitation training in school, as school hospital and college working together can realize resource sharing, introduce quality training resources, promote teachers to carry out CPR-related courses, and invite experienced medical and nursing staff to demonstrate operation and guidance, thus enhancing the training effect [5].

Training mode: Introduce the training mode, collect cases around college students, and make students realize that cardiac arrest not only happens in hospitals but can happen anywhere; make students realize the importance of mastering CPR-related knowledge; improve students' awareness of CPR knowledge; show relevant videos to students, where teachers demonstrate first aid techniques, and explain each step in detail. Students can discuss some of the details, perform first aid techniques, and compressions and exhalation on a simulator to make them feel it visually, and improve their awareness of first aid knowledge and master first aid operation techniques. Students can also be issued CPR-related manuals to facilitate random viewing [8].

To sum up, strengthening training on CPR-related knowledge for college students can improve their mastery of CPR knowledge and improve their ability to provide first aid.

## 5. Conclusion and Future Directives

To investigate the impact of holistic care on line coagulation and safety in hemodialysis, we proposed a combined deep learning approach for holistic care on line coagulation in hemodialysis. The velocity scales were first used to obtain the velocity along the sound beam direction provided by color Doppler echocardiography as the radial velocity component; then, the U-Net network was used to automatically identify the left ventricular wall contour and calculate the left ventricular wall velocity by retraining the PWC-Net model as the boundary condition of the continuity equation, and the velocity component of each blood mass in the vertical sound beam direction was obtained by solving the continuity equation (i.e. tangential velocity component); the nursing detail score, nursing attitude score, nursing professionalism score, and total satisfaction score of the study group were higher than those of the control group, and the differences were statistically significant (*P* < 0.05). Applying all-round nursing in hemodialysis can effectively reduce the incidence of line coagulation and complications, and improve the safety of hemodialysis, as well as improve patients' satisfaction with nursing care.

In future, we are interested in expending the operational capabilities of the proposed model along with the existing model to resolve various other issues that are tightly coupled with the healthcare sector.

## Figures and Tables

**Figure 1:** Schematic diagram of segmentation function of radial velocity and distance.

**Figure 2:** Schematic diagram of smoothing method.

**Figure 3:** U-Net model training and application process.

**Figure 4:** Schematic diagram of PWC-Net model structure.

**Figure 5:** Flow of left ventricular blood flow field visualization method.

**Figure 6:** Test image with color compensation results.

**Figure 7:** PWC-Net chamber wall displacement estimation results.

**Figure 8:** Comparison of speed vector map results.

**Figure 9:** Comparison of results of planar flow diagram.

**Table 1:** Summary information table of the ultrasound simulation dataset.

Dataset	Center frequency (MHz)	Sampling frequency (MHz)	Raw data size	Data logarithm
4 small sphere imitation data	5	40	2078 × 256	416
Complex breast structure data	5	40	3117 × 300	380

**Table 2:** Information on important training parameters of PWC-Net model.

Training phase	Training dataset	Number of iterations	Training strategy	Loss function
Phase I	4 small sphere imitation data	1200000	*S*_long_	L2l0ss + regular term
Phase II	Complex breast structure data	600000	*S*_fine_	L2l0ss + regular term

**Table 3:** Comparison of the incidence of pipeline coagulation and complications between two groups of patients [*n* (%)].

Group	*n*	Pipeline coagulation	Complication			
			Hemorrhage	Catheter infection	Left heart failure	Incidence rate
Control group	30	6 (20.00)	3 (10.000	4 (13.33)	2 (6.67)	9 (30.00)
Research group	30	1 (3.33)	1 (3.33)	1 (3.33)	0 (0.00)	2 (6.67)
*x* ^2^		4				5.455
		043				
*P*		0.044				0.020

**Table 4:** Comparison of nursing satisfaction scores between two groups ($\bar{x}\pm s$, points).

Group	*n*	Nursing details	Nursing attitude	Nursing professionalism	Total satisfaction
Control group	30	18.67 ± 4.52	19.06 ± 4.71	26.57 ± 5.13	72.39 ± 9.22
Research group	30	23.66 ± 4.67	24.02 ± 4.80	33.19 ± 5.29	89.57 ± 9.57
*x* ^2^		3.842	3.694	4.501	7.302
*P*		<0.05	<0.05	<0.05	<0.06

## Data Availability

The datasets used and analyzed during the current study are available from the corresponding author upon reasonable request.
